The article "Clinical Efficacy and Safety of Percutaneous Spinal Endoscopy versus Traditional Open Surgery for Lumbar Disc Herniation: Systematic Review and Meta-Analysis" was retracted in 2023. Reason: concerns about the peer review.

# Clinical Efficacy and Safety of Percutaneous Spinal Endoscopy versus Traditional Open Surgery for Lumbar Disc Herniation: Systematic Review and Meta-Analysis

**DOI:** 10.1155/2022/6033989

**Published:** 2022-03-16

**Authors:** Xingping Xu, Changwei Chen, Yong Tang, Fusheng Wang, Yangsheng Wang

**Affiliations:** ^1^Department of Orthopedics, 14F Yinzhou People's Hospital, No. 251 Baizhang East Road, Yinzhou District, Ningbo, Zhejiang Province, China; ^2^The Affiliated People's Hospital of Ningbo University, Ningbo, Zhejiang Province, China

## Abstract

**Objective:**

Systematic analysis of the incidence of percutaneous spinal endoscopic technique and traditional open surgery for lumbar disc herniation.

**Methods:**

A randomized controlled trial (RCT) and cohort study on complications related to traditional open surgery was searched on the MEDLINE, Cochrane Library, PubMed, Web of Science, Chinese journal full-text database (CNKI), Wanfang, and Embase database. Language is not limited. The quality of each study was evaluated, various complications were compiled into electronic baseline tables, and the data from these studies were available. Meta-analysis and synthesis were performed with the RevMan 5.3 software to evaluate the statistical significance of both surgical techniques in terms of various complications.

**Results:**

12 studies were eventually included, and a total of 2,797 patients were included in the analysis. Meta-analysis results showed that there was no statistical difference in postoperative paresthesia between percutaneous spinal endoscopy and traditional open surgery (OR = 1.17, 95% CI (0.82, 1.66), *P* = 0.38, *I*^2^ = 0%, *Z* = 0.88), direct nerve root damage (OR = 0.79, 95% CI (0.58, 1.07), *P* = 0.13, *I*^2^ = 73%, *Z* = 1.52), and intraoperative hemorrhage and hematoma formation (OR = 1.00, 95% CI (0.67, 1.48), *P* = 0.99, *I*^2^ = 0%, *Z* = 0.02), but there was a statistical difference in disc recurrence (OR = 2.24, 95% CI (1.56, 3.21), *P* < 0.0001, *I*^2^ = 81%, *Z* = 4.39).

**Conclusion:**

Compared with the traditional open surgical treatment of lumbar disc herniation, percutaneous spinal endoscopic technology has obvious advantages in reducing nerve root injury, dural injury, and surgical area wound complications, but it is limited to preventing the technical characteristics of the surgical site, which is worse than that of open surgery.

## 1. Introduction

With the development of the time, the continuous promotion of the concept of minimally invasive surgery and the rapid development of surgical instruments, the increasingly mature minimally invasive spine technology has begun to attract attention [1]. Xin et al. [2] has treated the lumbar disc herniation (percutaneous endoscopic lumbar decompression, PELD, with the use of a combined percutaneous spinal endoscopic system with wide-angle visual decompression in the disc with the help of arthroscopy). It has become one of the important means to treat lumbar disc herniation and lumbar degenerative diseases [3]. However, most previous surgeons remain more focused on technological reform and innovations, surgical techniques, and clinical efficacy. There are few studies on complications of surgery, and previous reports have only studied the treatment of the procedure for lumbar disc herniation alone [4]. With the continuous development of percutaneous spinal endoscopic technology and the continuous expansion of the treatment scope, the indirect decompression from endoscopic disc resection to the direct expansion of the spinal canal, lateral crypt, and nerve root canal is also changing accordingly. For each clinical surgeon, the complications of surgery are a great challenge, so it is only fully and systematically important to know and grasp the surgical complications. The common complications of PELD are summarized to provide a reference for clinical surgeons [5].

The article "Clinical Efficacy and Safety of Percutaneous Spinal Endoscopy versus Traditional Open Surgery for Lumbar Disc Herniation: Systematic Review and Meta-Analysis" was retracted in 2023. Reason: concerns about the peer review.

Postoperative sensory abnormalities are a specific and common complication of PELD, which is generally considered to be associated with the stimulation of the dorsal root ganglion (DRG) during surgery. Some scholars have also referred to it as the “solar burning syndrome,” with the incidence of about 2% to 17%. Kim et al. reported that with 93 laminina methods and 385 lamininal methods for lumbar disc disease, the incidences of postoperative sensory abnormalities were 16.13% and 7.53%, respectively. The reason may be caused by prolonged pulling stimulation of nerve roots during surgical operation [6]. Repeated positioning puncture, the use of microscopic abrasive, the use of ring saw and bone drilling for lamina and vertebral plate expansion, radiofrequency electrocoagulation, and rotation adjustment working casing to block the surrounding soft tissue may indirectly or directly stimulate the compression of nerve roots to make their ischemia and hypoxia and the corresponding symptoms. Anatomical changes in the lumbosacral nerve, lumbar trauma, and surgical history as well as foraminal size can also cause postoperative sensory abnormalities [7].

Most are because of direct damage to nerve roots during surgery and are one of the serious complications of PELD surgery. Cheng et al. [8] reported that the incidence of nerve root injury in 923 patients undergoing PELD for lumbar disc herniation was approximately 0.5%. Guo et al. [9] reported that the incidence of nerve root injury in 276 patients undergoing PELD for lumbar spinal stenosis was 1.1% [10]. The main reasons for its occurrence are summarized in the following points: anatomical structure factors, mainly including the anatomical variation in some patients and external physicians have an unclear understanding of the local anatomy, especially in the early stages of the technology, which eventually leads to nerve damage.

The article "Clinical Efficacy and Safety of Percutaneous Spinal Endoscopy versus Traditional Open Surgery for Lumbar Disc Herniation: Systematic Review and Meta-Analysis" was retracted in 2023. Reason: concerns about the peer review.

## 2. Materials and Methods

### 2.1. Search Strategy

This study was conducted according to the PRISMA systematic evaluation guidelines. Relevant meta-analysis and original literature were retrieved from the Medline, Cochrane Library, PubMed, Web of Science, Chinese journal full-text database (China National Knowledge Infrastructure, CNKI), Wanfang database, and Embase database. The time range is the library construction until November 2018. English retrieval keywords are Lumbar Discectomy Complication (s), Lumbar Discectomy Complication (s) and Outcome (s), and Lumbar and Discectomy or Percutaneous endoscopic lumbar discectomy and Complications (Figure 1).

### 2.2. Inclusion and Exclusion Criteria

1. Inclusion criteria: randomized controlled trial (RCT) and cohort studies on percutaneous endoscopic discectomy and traditional open discectomy for the treatment of lumbar disc herniation (LDH) which are not limited in language. Subjects: unlimited gender, age older than 18 years, diagnosed with single segment lumbar disc herniation by physical examination and imaging examination (CT and MRI) and ineffective after 3 months of conservative treatment. Intervention group (the percutaneous spinal endoscopic technical group): discectomy with the following characteristics was defined as the meridian: the cutaneous spinal endoscopic discectomy places the working sleeve directly into the disc or canal, combined with the percutaneous puncture technique and then uses the suction, grasping, electrocoagulation, and other techniques to remove the diseased part of the disc. The control group (the traditional open surgery group): traditional open laminectomy, lamenestration, hemilaminectomy, and translaminectomy discectomy.
2. Exclusion criteria: (1) randomized controlled trials (RCT) and cohort studies not related to the topic; (2) multisegment lumbar disc herniation, cauda equina syndrome, malignancy, spinal deformity, intervertebral hole injury, vertebral fusion, minimally invasive transabdominal and lumbar discectomy, and laminectomy; (3) preoperative studies with uncontrollable factors such as neurological injury, infection, or rheumatism; and (4) animal, in vitro, biomechanical studies were also excluded.

### 2.3. Evaluation of Literature Quality

The included literature was read in full and evaluated, and the disagreement is decided by discussion or by a third-party expert arbitration. Quality evaluation included in the RCT study was conducted according to the quality evaluation criteria recommended by the Cochrane system: (1) whether the randomization method is correct (selection bias); (2) adequate randomization concealment (selection bias); (3) whether the blinding method between participants and subjects is in place (implementation bias); (4) whether the blinding method of efficacy assessors is feasible (measurement bias); and (5) loss of visit. For the included observational studies and cohort studies, NOS can be used to evaluate the included studies. NOS adopts the semiquantitative principle of star system to make quantitative evaluation on the selection of research quality, comparability, and results (Figure 2).

The article "Clinical Efficacy and Safety of Percutaneous Spinal Endoscopy versus Traditional Open Surgery for Lumbar Disc Herniation: Systematic Review and Meta-Analysis" was retracted in 2023. Reason: concerns about the peer review.

### 2.4. Data Extraction and Analysis

Data were extracted and finally summarized and checked. Main observation indicators are total complications, postoperative sensory abnormalities (nerve root pain and burning nerve root pain), direct nerve root injury (any nerve root puncture or direct nerve root injury and nerve root displacement), dural injury (for perioperative dural damage and cerebrospinal fluid leakage), surgical area wound complications (including cellulitis, discitis, spondylitis, skin infection, superficial wound infection, suture granuloma, crack and hematoma), intervertebral disc recurrence (complete remission of nucleus removal after the same space ipsilateral or contralateral lumbar disc herniation, with radiographic confirmation), residual nucleus pulposus (no remission or incomplete postoperative symptoms, confirmed by review MRI as residual compression of the nerve root), additional surgery of related complications (secondary surgery due to disc recurrence, nucleus pulposus residual, or other related complications). Among them, it is difficult to analyze and obtain the small sample size and low incidence of events, which is difficult to obtain reference data, so it will be integrated into other complications for analysis and discussion. Using the Cochran database, the extracted data were analyzed by using the RevMan 5.3.0 software. A chi-square test was first used to determine the heterogeneity of each study result. There was significant interstudy heterogeneity when included at *P* < 0.1 or *I*^2^>50%. For those with heterogeneity, the causes of heterogeneity were first analyzed, and subgroup analysis and sensitivity treatment were conducted. If it has clinical consistency, the analysis was combined with a random effect model. Fixed-effect models were used for the study data without heterogeneity.

The article "Clinical Efficacy and Safety of Percutaneous Spinal Endoscopy versus Traditional Open Surgery for Lumbar Disc Herniation: Systematic Review and Meta-Analysis" was retracted in 2023. Reason: concerns about the peer review.

### 2.5. Bias Analysis

The data in this study were all dichotomous variables, and odds ratio (OR) and 95% confidence interval (CI) were calculated. If the analysis showed statistically significant differences in complications among studies, a funnel plot was used to analyze whether publication bias existed. Sensitivity analysis was performed on the effects of studies of low quality, particularly high weight or results that differed from other studies (Figure 3).

## 3. Result

### 3.1. Characteristics and Quality Evaluation of the Included Literature

The initial examination obtained 423 documents by reading text questions, abstract, and full text and finally included 24 relevant research articles, 12 randomized controlled trials and 12 cohort studies [11–22]. A total of 2,797 patients were included in this study. Basic characteristics of the included study are as follows: there were no significant baseline differences in gender or age of the patients included in the literature (Table 1). For the 12 cohort studies included, the NOS score was 5–9. For the 12 included randomized controlled studies, the Cochrane Risk of Bias tool was used for risk assessment.

### 3.2. Postoperative Paresthesia

Among the 4 RCT literatures included in percutaneous spinal endoscopy versus traditional open surgery for lumbar disc herniation, the heterogeneity test was carried out and it was found that the heterogeneity of the selected studies was small, so meta-analysis with fixed models could be performed. Meta-analysis results showed that there was no statistical difference in postoperative paresthesia between percutaneous spinal endoscopy and traditional open surgery (OR = 1.17, 95% CI (0.82, 1.66), *P* = 0.38, *I*^2^ = 0%, *Z* = 0.88) (Figure 4).

### 3.3. Direct Nerve Root Damage

Among the 4 RCT literatures included in percutaneous spinal endoscopy versus traditional open surgery for lumbar disc herniation, the heterogeneity test was carried out and it was found that the heterogeneity of the selected studies was small, so meta-analysis with fixed models could be performed. Meta-analysis results showed that there was no statistical difference in direct nerve root damage between percutaneous spinal endoscopy and traditional open surgery (OR = 0.79, 95% CI (0.58, 1.07), *P* = 0.13, *I*^2^ = 73%, *Z* = 1.52) (Figure 5).

### 3.4. Disc Recurrence

Among the 4 RCT literatures included in percutaneous spinal endoscopy versus traditional open surgery for lumbar disc herniation, the heterogeneity test was carried out and it was found that the heterogeneity of the selected studies was small, so meta-analysis with fixed models could be performed. Meta-analysis results showed that there was statistical difference in disc recurrence between percutaneous spinal endoscopy and traditional open surgery (OR = 2.24, 95% CI (1.56, 3.21), *P* < 0.0001, *I*^2^ = 81%, *Z* = 4.39) (Figure 6).

The article "Clinical Efficacy and Safety of Percutaneous Spinal Endoscopy versus Traditional Open Surgery for Lumbar Disc Herniation: Systematic Review and Meta-Analysis" was retracted in 2023. Reason: concerns about the peer review.

### 3.5. Intraoperative Hemorrhage and Hematoma Formation

Among the 4 RCT literatures included in percutaneous spinal endoscopy versus traditional open surgery for lumbar disc herniation, the heterogeneity test was carried out and it was found that the heterogeneity of the selected studies was small, so meta-analysis with fixed models could be performed. Meta-analysis results showed that there was no statistical difference in intraoperative hemorrhage and hematoma formation between percutaneous spinal endoscopy and traditional open surgery (OR = 1.00, 95% CI (0.67, 1.48), *P* = 0.99, *I*^2^ = 0%, *Z* = 0.02) (Figure 7).

## 4. Discussion

Surgical treatment of lumbar intervertebral disc herniation with the social development and scientific and technological progress has experienced from traditional to minimally invasive changes, and laminofenestration lumbar intervertebral disc resection is one of the classic traditional surgical treatments of LDH. Its clinical effect is satisfactory, but it causes lumbar rear muscle and bone structure damage, prone to lumbar instability and residual back pain [23]. At the same period, the technology was introduced into China, which favorably laid the foundation for the development of minimally invasive spine surgery technology in China. Wang et al. [24] invented the spinal endoscopic system (Thomas Hoogland Endoscopy Spine Systems, THESYS), which further developed as TESSYS. To enable the surgeon to reach the imaging and operating apparatus directly into the vertebral canal through the foramen to remove the protruding compressor, the technique is aided by a special multilayer drill hole which expands the foramen and the postoperative satisfaction rate can reach more than 80% [25]. However, in the process of TESSYS application in clinical practice, various complications such as inaccurate puncture positioning, medical personnel damage due to too long perspective time, damage to nerve roots and dura, long channel establishment time, and other problems often occur. However, with the continuous development of percutaneous spinal endoscopic technology and the improvement of instruments, the efficacy and safety in the treatment of lumbar disc herniation are continuously improved [26].

Transcutaneous spinal endoscopic technology for lumbar disc herniation compared with traditional open surgical technology: its advantages are recognized by scholars, but its surgical complications are controversial. This study analyzed the percutaneous spinal endoscopic technology and traditional open surgery treatment of the LDH trial and cohort study [27], and the results show that the former in the total complications, direct nerve root injury, dural sac injury, and surgical wound complications were significantly better than the latter and in the myeloid residue inferior to the latter [28]. The results also showed no significant differences among the two technical methods in postoperative sensory abnormalities, disc recurrence, or other complications. Some scholars [29] believe that percutaneous spinal endoscopic technology after percutaneous puncture positioning casing and endoscopy directly by the foraminal area into the spinal canal and in the circulating water environment avoid large incision exposure, and timely debris, intraoperative bleeding point in the intraoperative area clearly visible, plasma bipolar radiofrequency hemostasis, and various conditions reduce the surgical area wound complications [30].

The article "Clinical Efficacy and Safety of Percutaneous Spinal Endoscopy versus Traditional Open Surgery for Lumbar Disc Herniation: Systematic Review and Meta-Analysis" was retracted in 2023. Reason: concerns about the peer review.

The total incidence of complications varied between the two surgical techniques in this study; however, due to the high heterogeneity, a subgroup analysis was performed and the results showed that percutaneous spinal endoscopic techniques outperform traditional open surgery in total complications. Also, it has statistical significance. However, percutaneous cohort endoscopy and traditional open surgery did not show significant advantages and disadvantages in the cohort study. The reason may be the large reporting bias in observational studies, leading to greater heterogeneity in the study. Due to the great controversy between the two techniques in postoperative disc recurrence, this study is hereby conducted according to the follow-up time subgroup analysis, and the results indicated no statistically significant complication incidence of postoperative disc recurrence between the two techniques.

The limitations of this study are as follows: (1) incorporating observational studies in the study is limited; (2) the follow-up varies from 3 to 36 months, making the evaluation of long-term complications; (3) the publication bias analysis is only qualitative and large personal factors; and (4) the two techniques described in this paper contain multiple surgical procedures, which may increase the bias of the study. Since the assessments were all based on a small number of studies, the results must be interpreted with caution. As the accumulated evidence grows, our conclusions may either be supported or overturned.

Compared with the traditional open surgical treatment of lumbar disc herniation, percutaneous spinal endoscopic technology has obvious advantages in reducing nerve root injury, dural injury, and surgical area wound complications, but it is limited to preventing the technical characteristics of the surgical site, which is worse than that of open surgery.

The article "Clinical Efficacy and Safety of Percutaneous Spinal Endoscopy versus Traditional Open Surgery for Lumbar Disc Herniation: Systematic Review and Meta-Analysis" was retracted in 2023. Reason: concerns about the peer review.

## Figures and Tables

**Figure 1:** Flow chart of the literature screening.

**Figure 2:** Literature quality evaluation chart. (a) Risk of bias graph. (b) Risk of bias summary.

**Figure 3:** (a, b) Funnel plot of literature publication bias.

**Figure 4:** Meta-analysis of postoperative paresthesia between two groups.

**Figure 5:** Meta-analysis of direct nerve root damage between two groups.

**Figure 6:** Meta-analysis of disc recurrence between two groups.

**Figure 7:** Meta-analysis of intraoperative hemorrhage and hematoma formation between two groups.

**Table 1:** Basic clinical features of 12 literatures included in our study.

Study	Age	Gender (man)	Experimental group (N)	Control group (N)	NOS score	Research type	*P* values of HWE
Heo et al. (2019) [11]	43.71 ± 12.2	45.25	96	75	8	RCT	0.35
Cheng and Chen (2020) [8]	45.65 ± 13.4	59.12	86	63	8	RCT	0.02
Lohre et al. (2020) [12]	62.12 ± 14.5	55.72	118	108	8	RCT	0.04
Carbó et al. (2019) [13]	57.15 ± 14.5	54.12	66	60	7	RCT	0.12
Wu et al. (2020) [4]	52.45 ± 8.4	54.89	58	73	8	RCT	0.06
Yang et al. (2020) [14]	64.26 ± 10.2	53.45	54	65	7	RCT	0.02
Ao et al. (2020) [15]	62.45 ± 12.2	48.10	80	75	9	RCT	0.01
Li et al. (2020) [16]	62.51 ± 13.0	58.75	80	63	8	RCT	0.02
Feng et al. (2020) [17]	47.25 ± 14.5	55.23	41	56	7	RCT	0.14
Li et al. (2020) [18]	56.22 ± 15.2	46.22	64	70	8	RCT	0.23
Wang et al. (2021) [19]	51.35 ± 8.1	54.16	108	100	7	RCT	0.01
Yu et al. (2020) [20]	57.65 ± 16.0	56.34	96	77	7	RCT	0.25

## Data Availability

The data used to support the findings of this study are available from the corresponding author upon request.
